# Protective Effect of Melatonin on Nonylphenol-Induced Reproductive and Behavioral Disorders in First-Generation Adult Male Rats

**DOI:** 10.1155/2022/1877761

**Published:** 2022-04-26

**Authors:** Mahsa Tavakoli, Ali Akbar Moghadamnia, Fereshteh Pourabdolhossein, Mohammad Hossein Asghari, Sohrab Kazemi

**Affiliations:** ^1^Student Research Committee, Babol University of Medical Sciences, Babol, Iran; ^2^Department of Pharmacology and Toxicology, School of Medicine, Babol University of Medical Sciences, Babol, Iran; ^3^Cellular and Molecular Biology Research Center, Health Research Institute, Babol University of Medical Sciences, Babol, Iran; ^4^Neuroscience Research Center, Health Research Institute, Babol University of Medical Sciences, Babol, Mazandaran, Iran

## Abstract

**Methods:**

Pregnant Wistar rats were randomly assigned into five groups: control, NP (25 mg/kg), NP (25 mg/kg)+MLT (10 mg/kg), NP (25 mg/kg)+MLT (20 mg/kg), and MLT (20 mg/kg). The duration of treatment was 21 days from gestation time. Morris water maze was used to assess learning and memory. NP concentrations of serum and testicular tissue were measured by HPLC. Histological analysis of testicular tissues was done by H&E staining.

**Results:**

Behavioral study showed that NP does not impair learning and memory in first-generation rats. Histomorphometric results showed that NP can significantly reduce the cross-sectional area of the seminiferous tubules and the epithelium, the diameter and number of seminiferous tubules, the thickness of the epithelium, and the number of spermatocytes and spermatogonia compared to other groups. MLT reversed the NP-induced histomorphometric. Also, it changes and increased the activity of superoxide dismutase (SOD), total antioxidant capacity (TAC), and catalase (CAT). The level of malondialdehyde (MDA) significantly decreased in MLT-treated groups compared with the NP group.

**Conclusion:**

Our finding showed that MLT enhanced the learning process and reduced NP-induced testicular tissue damage through its antioxidants and cytoprotective effects.

## 1. Introduction

NP has been widely used as wetting agents, detergents, and emulsifiers in industry and is also present in household toiletries, paints, and pesticides [1]. NP as an endocrine disrupting chemical (EDC) could play an important role in the production of free oxygen radicals. Free oxygen radicals cause an increase and decrease in the levels of malondialdehyde (MDA) and glutathione (GSH), respectively. NP could have adverse effects on health including the reproductive and central nervous system (CNS) [2, 3]. The previous studies have suggested that NP could impact the reproductive system by inducing oxidative stress and decreasing the activity of scavenging enzymes, glutathione peroxidase, and superoxide dismutase in the testis tissue. Several lines of evidences proved that NP exposure caused reduction of sperm counts and epididymal weights [4], decreased the number of germ and Sertoli cells, diminished weight/volume of the testis [5], and impaired sperm function and motility [6]. Moreover, NP-induced oxidative stress contributes to cytotoxicity through apoptosis in neural stem cells, which suggests that NP might affect neurogenesis in the CNS [2]. It has been suggested the NP directly or indirectly is involved in the pathogenesis of neuropsychiatric disorders such as attention deficit hyperactivity disorder (ADHD) and autism due to the dysfunction of dopaminergic and other neurotransmitter systems in CNS [1].

MLT, a tryptophan-derived neurohormone, is mainly produced by the pineal gland and mediates its effects by binding to MLT receptor type 1 (MT1) and 2 (MT2) [3]. MLT has numerous effects on the release of gonadotropins by the anterior pituitary, as well as on gonads and gonadal adnexa since its specific receptors are widely distributed throughout the reproductive tract [4, 5]. MLT possesses antioxidant with prophylactic characteristics against oxidative stress [5, 6]. Free-radical scavenging property of MLT might protect against the adverse effects of EDCs on testicular function and spermatogenesis due reducing oxidative damage and controlling the levels of the antioxidant enzymes [7–11]. Previous reports have demonstrated that antioxidants such as lipoic acid [12], N-acetylcysteine [13], vitamin C [14], and gallic acid [15] could prevent or reduce the EDC-induced toxicity effects. The ameliorative role of MLT has been reported in EDC-induced biochemical toxicity in testicular mitochondria of adult mice [16].

A recent study on the importance of MLT roles on the CNS has implied its protective roles in the CNS by inducing the proliferation, differentiation, and survival of neural cells. Moreover, MLT prevents neural cells from potentially excessive glucocorticoids, hypoxia, and inflammation [17]. Thus, the present study was designed to investigate the protective effect of MLT on reproductive and behavioral dysfunction induced by NP in first-generation adult male rats.

## 2. Materials and Methods

### 2.1. Chemicals

NP (>99% pure) and MLT as powder (≥98% purity) were purchased from Kento, Japan, and Sigma-Aldrich (St. Louis, Mo, USA), respectively. NP was dissolved in soya oil as a vehicle. MLT was daily completely mixed with distilled water by an ultrasonic homogenizer.

### 2.2. Experimental Groups and Intervention

The pregnant female rats (weighing 150–200 g) were obtained from the Babol University of Medical Sciences' Animal room (Babol, Iran). All rats were kept in plastic cages under controlled light and dark conditions (12 h light : 12 h dark) at 22 ± 2°C and humidity of 50 ± 5%, with free access to chow and tap water *ad libitum*. All the experiments were performed in accordance with the international guidelines for the safe working of animals, and the project was approved by the Babol University of Medical Sciences Ethics Committee (IR.MUBABOL.REC.1399.002).

Pregnant rats were assigned into five groups (*n* = 3):

1. Control (soy oil receiving by gavage)
2. NP (25 mg/kg, by gavage)
3. NP (25 mg/kg, by gavage)+MLT (10 mg/kg, IP)
4. NP (25 mg/kg, by gavage)+MLT (20 mg/kg, IP)
5. MLT (20 mg/kg/IP)

All treatments were given for 21 days during gestation time. After birth and lactation, male pups were kept in separate cages until puberty (*n* = 8). Morris water maze test was performed for adult male rats (age 2 months). The rats were then anesthetized using ketamine (10%) and xylazine (2%), and the testes were removed and stored for histopathological and histomorphometry evaluation. The blood samples were taken and stored at -80°C for assessment of the level of NP, MLT, testosterone, and antioxidant enzymes.

### 2.3. Morris Water Maze Test

The Morris water maze test was performed as described by Lu et al. [18]. The experimental apparatus consisted of a circular water tank (100 cm in diameter, 35 cm in height), containing water (23 ± 1°C) to a depth of 15.5 cm, which was rendered opaque by adding ink. A platform (4.5 cm in diameter, 14.5 cm in height) was submerged 1 cm below the water surface and placed at the midpoint of one quadrant. The pool was located in a test room, which contained various prominent visual cues. Each rat received four training periods per day for 4 consecutive days. The training was such that first the rats of a group were released from the first quadrant of the tank and trained. The rats were then released from the second quadrant and trained again. This rhythm continued until the end of the 4 quadrants, and the same continued until the training of all 5 groups. Latency to escape from the water maze (finding the submerged escape platform) and swimming distance and the swimming speed were analyzed to assess spatial learning. To evaluate the spatial memory, on day 5, the probe test was carried out by removing the platform and allowing each rat to swim freely for 60 s. The times that rats spent swimming in the target quadrant (where the platform was located during hidden platform training) were measured. EthoVision XT 11 software (Noldus, Netherlands) was used to capture and analyze the mentioned parameters.

### 2.4. Preparing the Blood Samples

Blood samples (2 ml) were obtained by cutting the auxiliary artery for each adult male rat and were transferred into 5 ml tubes. Then, the samples were separately centrifuged and the serums were kept at −80°C for further analysis.

### 2.5. Testosterone (Serum) Assay by ELISA

The level of testosterone was measured using an ELISA kit made by Demeditec Company (Germany). Frozen stored serum samples were allowed to thaw at room temperature. They were then centrifuged at 2500 rpm for 15 min. The optical densities of the samples containing testosterone were measured using an ELISA reader (Rayto microplate RT-2100C) at wavelengths of 450 and 630 nm [19].

### 2.6. Biochemical Assays (Oxidative Parameters)

Antioxidant and oxidant markers including superoxide dismutase (SOD), catalase (CAT), total antioxidant capacity (TAC), and malondialdehyde (MDA) were detected by Razi Medical Research Company Kits (Iran).

### 2.7. Determination of Serum SOD Activity

Superoxide dismutase enzyme activity was assayed using the method of Peltola et al. [20]. SOD activity is measured using tetrazolium salt, which produces a water-soluble dye by reducing the superoxide anion. The formation rate of formazan is inhibited by the presence of SOD in the environment and can be measured photometrically. Serum SOD was measured at 440 nm and reported as units per milliliter.

### 2.8. Determination of Serum CAT Activity

CAT activity was assayed by the method of Aebi [21]. The catalase activity was calculated by an ELISA reader at 540 nm, in terms of nmol H_2_O_2_ consumed min.

### 2.9. Determination of Serum TAC Activity

The TAC of plasma was measured according to the method of Güney et al. [22]. The kit used to measure TAC uses a chromogenic peroxidase substrate, which produces a water-soluble chromogen upon oxidation by ferryl myoglobin radicals. The green chromogen formation rate is inhibited by the presence of antioxidants in environments. TAC was measured at 412 nm by an ELISA reader.

### 2.10. Measurement of Serum Malondialdehyde (MDA)

The concentration of MDA in serum was determined as thiobarbituric acid reactive substances (TBARS) according to and as described by Placer et al. [23]. Teb Pazhouhan Razi Assay Kit was used for this assay, and the results were expressed as micromolar.

### 2.11. Histopathology and Morphometric Studies

The left testis of each rat was collected then fixed in 10% formalin. After one week of fixation and processing of samples by the conventional methods, paraffin sections were obtained. The embedded paraffin sections were cut at 5 *μ*m then stained by H&E staining method for histopathological examination. Microscopic grading and scoring of the testis tissue sections were carried out to determine the degree of severity of the observed histopathological lesions according to Hassanen et al. [24]. Grading of damage was performed according to the following parameters: tissue swelling, necrosis, fibrosis, the rate of destruction of spermatozoa, hyaline deposition, destruction of the basement membrane in spermatozoa, and changes in the size and shape of tissue cells. The above parameters were assessed and scored as mild, moderate, and severe, as follows: (−) normal histology; (+) mild <25%; (++) moderate 25–50%; and (+++) severe >50% of the tissues affected.

### 2.12. Histomorphometry

The histomorphometric examination was performed as we previously described [25]. Figures were obtained from the smears using an Olympus optical microscope equipped with a Canon camera at a magnification of 10x, and 40x at four random points, and a TCapture software made by Chinese company TUCSEN application was used for extracting the data.

### 2.13. Measurement of Seminiferous Tubule Diameter

For each animal, 10 seminiferous tubules were randomly chosen from figures with a magnification of 10x, and for each tubule, long diameters were measured. The data were analyzed using statistical tests.

### 2.14. Thickness of Epithelium of Seminiferous Tubules

The thickness of the epithelium of the seminiferous tubules was measured in five groups. The heights of the epithelium for 100 tubules in four directions and four angles were measured.

### 2.15. Surface Area and Cross-Sectional Area of the Epithelium of Seminiferous Tubules

The cross-sectional area of seminiferous tubules was measured and recorded using TCapture software. Also, the lumen area of the seminiferous tubules was measured. Then, by subtracting these two numbers from each other, the cross-sectional area of the epithelium of seminiferous tubules was calculated. The same tubules are used to reduce the error in all of the above cases.

### 2.16. Number of Seminiferous Tubules

For each rat, 40 figures with a magnification of 10x were chosen. For an accurate recording, a square with an area of 5.3302 cm^2^ was drawn. All tubules in the middle and on the top right of the square were counted. Then, the number of seminiferous tubules was divided by the square area (5.3302 cm^2^) to obtain the number of seminiferous tubules in 1 cm^2^.

### 2.17. Number of Spermatocytes and Spermatogonia

For each rat, 4 figures with a magnification of 40x were chosen. First, the area of the seminiferous tubule was calculated using a TCapture software. Then, the number of spermatogonia, which looked round with dark circles in the outer layer of the epithelium, was counted. In the next step, the number of spermatocytes was recorded. Finally, the number of spermatocytes and spermatogonia was divided by the area of the seminiferous tubule to obtain the number of spermatocytes and spermatogonia per unit area.

### 2.18. Measurements of NP in Serum and Testis Tissue by HPLC

The HPLC (KNAUER Co, Germany), consisting of a C18 column and a fluorescence detector (Shimadzu, Japan) set at an excitation wavelength of 227 nm and an emission wavelength of 313 nm was used. Mobile phase A was acetonitrile, and mobile phase B was water. The system was run in a linear gradient: 0–6.0 min A 70%, B 30%; 6.0–6.2 min mobile phase A increased from 70 to 100% and continued to minute 12. The chromatographic analysis was performed at 25°C with a flow rate of 0.8 ml/min and an injection volume of 20 *μ*l. Data collection was accomplished using EZChrom software and finally was statistically analyzed.

## 3. Serum and Tissue Sampling

### 3.1. Extraction of Serum Sample

One hundred microlitres of 0.01 mol/l ammonium acetate buffer (pH 4.5) and 4 ml mixed solvent of n-hexane and diethyl ether (70 : 30, *v*/*v*) were added to 500 *μ*l of serum. The samples were centrifuged, and the organic layer was evaporated to dry the sample under gentle nitrogen flow. The samples were reconstituted with 100 *μ*l of acetonitrile for analysis [26].

### 3.2. Extraction of Tissue Samples

Extraction of samples was done by the method of Xiao et al. [26]. The testis tissue (200 mg) was accurately weighed. The samples were homogenized with 2.0 ml of 0.01 mol/l ammonium acetate buffer (pH 4.5) for 1 min at room temperature. Methanol (8.0 ml) and 100 *μ*l of perchloric acid (4.0 mol/l) were added to the homogenate. The sample was agitated on a vortex mixer, sonicated for 10 min, and centrifuged for 10 min at 12.000 rpm (Polish MPW Company). The supernatant of 5.0 ml was taken to a glass tube, to which 0.01 mol/l of ammonium acetate buffer (pH 4.5) was added up to 20 ml and mixed to yield a solution. The C18 SPE cartridge (INOPAK) was conditioned with 10 ml of methanol and equilibrated with 5 ml of water and 5 ml of 0.01 mol/l ammonium acetate buffer (pH 4.5) prior to use. Then, the sample solution was loaded to the cartridge, washed with 5 ml of water (residual water was removed by placing the cartridge under vacuum for 30 s), and eluted with 4.0 ml of methanol at a low flow rate (1 ml/min). If the sorbent in the cartridge runs dry any time before the sample-loading step into the cartridge, the consequence is low and variable recovery. The eluting solution was evaporated to dry the sample with a rotary-vacuum evaporation apparatus at 45 ± 1°C and reconstituted in 100 *μ*l of acetonitrile. The obtained samples were analyzed by HPLC.

### 3.3. Statistical Study

All data were analyzed using GraphPad Prism 6. The experimental results are expressed as mean ± SD. Behavioral data from the training period were analyzed using repeated measure two-way ANOVA followed by Tukey post hoc test. The data from probe test, histology, and biochemical assays were analyzed by one-way ANOVA followed by post hoc Tukey test. The differences between data of the groups were assumed significant at *p* < 0.05.

## 4. Results

### 4.1. Morris Water Maze Test

The Morris water maze test was used to evaluate the effects of NP and MLT treatments on learning and memory function. No significant delay was observed in the time to reach the platform during training trials (day 1 to 4) in the NP-treated group compared with the control. The escape latency to find the hidden platform was significantly decreased in the NP+MLT10 group on days 1 and 2 compared to the control (*p* < 0.001), NP (*p* < 0.0001), NP+MLT20 (*p* < 0.001), and the MLT20 (*p* < 0.01) groups. In comparison within the control group, escape latency was significantly decreased at day 4 (*p* < 0.0001) and day 3 (*p* < 0.0001) compared to day 1 and day 2 (*p* < 0.001and *p* < 0.01), respectively. Moreover, in the NP25 group, this significant decrease was observed at days 3 and 4 compared to days 1 and 2 (*p* < 0.05). In comparison within the NP+MLT10 group, escape latency was significantly reduced at days 3 and 4 (*p* < 0.01) and day 2 (*p* < 0.005) compared to day 1. Also, in the NP+MLT20 group, escape latency significantly decreased on day 4 compared with days 1 (*p* < 0.0001) and 2 (*p* < 0.01) and day 3 compared to day 1 (*p* < 0.0001) and day 2 (*p* < 0.005) (Figure 1(a)). Furthermore, in the MLT20 group, escape latency on days 3 and 4 markedly decreased compared with day 1 (*p* < 0.0001) and day 2 (*p* < 0.001). In comparison between groups only in the NP+MLT10 group, we observed a significant difference in training trails (Figure 1(a)).

Data from distance moved in training trails was compatible with escape latency, and no significant differences were observed between the NP-treated group and control in all training days which confirmed learning was not affected in NP groups. In the NP+MLT10 group, the distance moved to reach the platform was significantly decreased on day 2 (*p* < 0.0001) and 1 (*p* < 0.01) compared with the control group and on day 2 (*p* < 0.0001) compared to the NP-treated group. Also, in the NP+MLT10 group, the distance traveled to reach the platform markedly decreased on days 1 and 2 (*p* < 0.0001) compared to the NP+MLT20 group and days 1 (*p* < 0.0001) and 2 (*p* < 0.001) compared to the MLT20 group (Figure 1(b)).

Swimming speed did not show a significant difference between all groups, so NP and MLT had no effect on motor activity and animal speed. This confirms that there is no movement disorder in this model (Figure 1(c)).

For assessment of spatial memory, at the last day of the experiment (day 5), the platform was removed and the time spent in the target quadrant was analyzed as a spatial memory index in all experimental groups. Tukey post hoc analysis showed that the time spent in the target quadrant in the NP25 group was not significantly different with control and MLT-treated groups. Therefore, NP as well as MLT in different doses in mothers had no effect on the spatial memory of first-generation animals (Figure 1(d)).

### 4.2. MLT Modulated Oxidative and Antioxidant Factors

Catalase activity in NP25 group noticeably decreased compared to the control and MLT20 groups (*p* < 0.05) (Figure 2(a)). The mean concentration of MDA in the NP25 group was markedly higher than that in control group (*p* = 0.0003). The MDA in the NP+MLT10 (*p* = 0.0002), NP+MLT20 (*p* < 0.0005), and MLT20 (*p* < 0.001) groups was significantly decreased compared with that in the NP25 group (Figure 2(b)). The mean total antioxidant capacity (TAC) in the NP25 group was significantly lower than that in the control group (*p* < 0.001). The mean TAC in the NP+MLT20 group (*p* = 0.03) and the MLT20 group (*p* < 0.001) was markedly increased compared with that in the NP25 group (Figure 2(c)). Moreover, superoxide dismutase activity in the NP25 group was significantly lower than that in the control group (*p* < 0.001). The SOD activity was noticeably increased in the NP+MLT10 (*p* = 0.03) and MLT20 (*p* = 0.003) groups compared with the NP25 group (Figure 2(d)).

### 4.3. Change in Serum Hormone Level

The levels of testosterone are slightly, but not significantly, lower in the NP25 group compared to the control and the other groups (Figure 3).

## 5. HPLC Assay

### 5.1. Serum and Tissue Concentration of Nonylphenol

To determine the concentration of NP in serum and testicular using HPLC method, the mean and standard deviation of NP concentrations were measured, and there were significant concentrations in the testicular tissues of rats in the NP group compared to treatment groups (*p* < 0.05) (Table 1). The concentrations of NP in the serum and testicular tissues were determined based on the internal standard method using calibration curves. The calibration curves are presented in Figure 4.  Figure 5 (chromatogram) also shows sample HPLC chromatograms obtained for NP analysis.

### 5.2. Morphometric Findings in Testicular Tissue

The mean of the diameters of the seminiferous tubules and the mean of the four heights drawn for the epithelium of the seminiferous tubules for all groups were calculated. The highest diameter and thickness of epithelium of the seminiferous tubules belonged to the control group and the least to the NP25 group. No significant difference was observed in the diameter of the seminiferous tubules between the all groups of the study.

A significant decrease was noted in the thickness of the epithelium in the NP receiving group compared to the control and the MLT20 groups (*p* < 0.05). The cross-sectional and surface area of the epithelium of the seminiferous tubules was calculated and is shown in Table 2. The highest cross-sectional area of seminiferous tubules and the epithelium belongs to the MLT20 group, and the lowest was shown in the NP-treated group.

The cross-sectional area of the seminiferous tubules in the NP group was significantly decreased compared with all groups. The surface area of the epithelium of the seminiferous tubules in the control group and the MLT20 group showed a significant difference compared to the NP group and NP+MLT10 group and NP+MLT20 group (*p* < 0.05). The mean (±SD) of surface of seminiferous tubules is presented in Table 2, with the highest surface shown in the control group, and the lowest is belonging to the NP group. There was a significant decrease in the number of seminiferous tubules between the NP25 group and other groups (*p* < 0.05). The number of spermatocytes and spermatogonia in the seminiferous tubules was counted. Table 2 shows the mean (±SD) of the number of spermatocytes and spermatogonia. The highest number of spermatogonia was in the control group and the highest number of spermatocytes in the MLT20 group, whereas the lowest number belonged to the NP25 group. Statistical analyses showed that the number of spermatocytes in the NP25 group significantly decreased compared with all groups. Moreover, the number of spermatogonia in the NP25 and NP+MLT10 groups significantly decreased compared to that in other groups (*p* < 0.05).

### 5.3. Histopathological Changes of Testicular Tissue

The microscopic images of the testicular cross-section of the rats showed that the testicular tissue in the control (Figure 6(a)) and MLT 20 (Figure 6(b)) groups was in normal condition. Also, in the MLT20 group, we found a normal pattern of spermatogenic cells in the seminiferous tubules and an increase in the spermatozoa population. In the NP25 group, hyperemia, edema, vacuolar degeneration, and disruption in the germinal tissue of seminiferous tubules were observed which is characterized by the loss of germinal tissue cohesion and creating a gap between them and spermatozoa population was decreased (Table 3) (Figure 6(c)). However, MLT treatment in the NP+MLT10 (Table 3) (Figure 6(d)) and NP+MLT20 (Table 3) (Figure 6(e)) groups enhanced the repair of the germinal tissue of seminiferous tubules.

## 6. Discussion

We found that NP does not affect the learning and memory function in first-generation adult male rats. However, NP induced oxidative stress through enhancing MDA and reducing total antioxidant capacity and antioxidant enzymes. Histopathological results confirmed that NP induced hyperemia, edema, vacuolar degeneration, and disruption in the germinal tissue of seminiferous tubules and reduced spermatozoa, spermatocytes, and spermatogonia population. The present study presented that MLT at dose 10 mg/kg treatment enhanced learning process compared with other groups. Moreover, MLT reduced MDA as an oxidative factor and increased TAC and SOD. Finally, MLT improved the histopathological changes induced by NP in a dose-dependent manner. Thus, MLT cytoprotective and antioxidant properties could be beneficial for the treatment of NP-induced toxicity.

Here, we found that NP at dose 25 mg/kg had no effect on learning (escape latency and distance moved) and memory (time spent in target quadrant) in first-generation male rats. Jie et al. [1] reported that NP at a dose of 200 mg/kg reduced learning and memory function in first-generation male rats. It has also been reported that NP exposure at dose 100 mg/kg for 21 days of gestation reduced memory and learning in first-generation male rats [27]. The inconsistency of our results with aforementioned studies might be due to different doses of NP. It was proved that NP increases the expression of the glial fibrillary acidic protein (GFAP) as a specific astrocyte marker and as a result, it changed the morphological structure of astrocytes and causes apoptosis of neurons in the hippocampus, leading to learning and memory impairment [28].

We found that NP caused histopathological changes such as vacuolar degeneration, edema, and disruption in the germinal tissue of seminiferous tubules. It also reduced the cross-sectional area of seminiferous tubules and seminiferous tubule epithelium, the diameter and number of seminiferous tubules, the thickness of the epithelium, and also number of spermatocytes, spermatogonia, and spermatozoa population. In consistent with our findings, several studies showed that oxidative stress caused by NP is the main reason of damage to the reproductive system [29–34]; NP increases the production of free radicals and reduces the activity of antioxidant enzymes which induces oxidative stress in testicular tissue. Testicular organs have high metabolic rate and cell proliferation; therefore, the balance of free radicals and antioxidant enzymes in this tissue is very important. Disturbance of oxidant/antioxidant balance in the testicular tissue disrupted the key processes such as spermatogenesis. Moreover, oxidative stress leads to tissue damage, germ cell death, and impaired spermatogenesis [35].

Previous studies have shown that exposure to NP by increasing reactive oxygen species (ROS) and decreasing the activity of antioxidant enzymes including superoxide dismutase (SOD), glutathione reductase (GRD), and glutathione peroxidase (GPX) induces oxidative injury [27]. In line with these studies, our results showed that NP, by inducing lipid peroxidation, increased the concentration of MDA and decreased the SOD and catalase activity and total antioxidant capacity.

In this study, MLT was used as a potent antioxidant against the destructive effects of NP. It has been found that MLT has the ability to penetrate all cells of the body and neutralize free radicals [36].

It also increases the expression or activity of antioxidant enzymes such as SOD, CAT, and glutathione peroxidase through MT1 and MT2 membrane receptors and reduces oxidative stress [37]. Our behavioral data showed that MLT at a dose of 10 mg/kg enhanced the learning compared with NP25 and control groups and has a positive effect on the learning process. Soleimani et al. [37] showed that MLT is effective and has a protective effect on learning at dose 10 mg/kg in first-generation male rats. Correspondingly, a study by Baydas et al. [38] showed that coadministration of MLT with alcohol for 45 days was effective and improved alcohol-induced spatial learning and memory disabilities in rats. Another study by Tabassum et al. [39] examined the antioxidant effects of MLT on adult male rats exposed to NP and reported that MLT at dose 10 mg/kg improved learning and memory. MLT improves oxidative stress damages caused by NP through its potent antioxidant property.

Our histopathological data showed that MLT reduced the histopathological changes induced by NP in a dose-dependent manner. We showed that the antioxidant effect of MLT at dose 20 mg/kg improved the histomorphometrical changes induced by NP and increased the spermatozoa population. MLT also improved vacuolar degeneration, edema, and disruption in the germinal tissue of seminiferous tubules. Previous studies have been shown that MLT with its antioxidant properties prevents oxidative stress, improves the morphology of seminiferous tubules, and inhibits apoptosis of germ cells [40]. The cytoprotective effects of MLT have been reported in cadmium chloride-induced toxicity in seminiferous tubules [41]. Moreover, it was shown that MLT prevents spermatocyte and spermatid loss caused by cyclophosphamide [11].

Our biochemical studies proved that MLT treatment at doses 10 and 20 mg/kg increased the activity of antioxidant enzymes and total antioxidant capacity in the NP-treated groups. Moreover, MLT reduced MDA as marker of lipid peroxidation. In line with our results, Sarabia et al. [42] showed that rats treated with MLT (10 mg/kg) and diazinon have lower concentration of MDA. It was also shown that coadministration of MLT with cadmium during the prenatal and postnatal period increases the activity of CAT and superoxide dismutase enzymes and decreases the concentration of MDA compared to the cadmium group [43].

Testosterone levels did not change in the NP, control, NP+MLT10, NP+MLT20, and MLT20 groups. However, Nagao et al. [44] found that NP decreased the testosterone levels. It was reported that NP has antiandrogenic effects; it induced oxidative stress and reduced the levels of enzymatic and nonenzymatic antioxidants in the Leydig cells which lead to testosterone reduction [33]. In another study, it has been shown that combined treatment with MLT and busulfan increased testosterone levels compared with busulfan alone [45]. Further studies are needed to understand the exact mechanisms of MLT and NP on testosterone secretion.

The NP concentration was measured using the HPLC with fluorescence detector. HPLC assay results in the present study showed that the highest concentration of NP in the serum and testicular tissue was reported in the NP group, although the measured concentration of NP was directly related to the dose consumed but did not affect the learning and memory function in first-generation adult male rats. However, oxidative stress and histopathological changes were seen in the testicular tissue such as vacuolar degeneration, edema, and disruption in the germinal tissue of seminiferous tubules, and these results were consistent with the results of a study by Soleimani et al. [37].

## 7. Conclusion

Our study discovered new insights into the efficacy of MLT on oxidative injury induced by NP toxicity. We found that MLT at dose 10 mg/kg enhanced learning in NP-treated groups. Moreover, MLT neutralized oxidative stress which can lead to inflammation and subsequent histopathological lesions. MLT has a protective effect on the reproductive system of male rats by increasing the number of sperm, reducing hyperemia, and vacuolar degeneration. Its antioxidant property has beneficial effects on the nervous system. Further studies are required to evaluate the potential benefits and underlying mechanisms of MLT on NP-induced toxicity.

## Figures and Tables

**Figure 1:** NP did not affect learning and memory in the first generation of adult rats but MLT improved learning. Comparison of mean (a) escape latency, (b) distance traveled to reach the platform, (c) swimming speed from day 1 to day 4 of training trial, and (d) time spent in the target quadrant in the probe trial in the Morris water maze test. A, B, C, D, and E: comparison within groups. ^∗∗∗∗^*p* < 0.0001, ^∗∗∗^*p* < 0.001, ^∗∗^*p* < 0.01, and ^∗^*p* < 0.05: comparison in between groups. Data from training trials were analyzed by repeated measure two–way ANOVA and probe test with one-way ANOVA coupled with Tukey post hoc test. Data are presented as means ± SD for eight animals in each group.

**Figure 2:** MLT balanced oxidative and antioxidant mediators in NP-treated rats. Comparison of (a) catalase activity, ^∗^significant difference from the control group at *p* < 0.05; ^++^significant difference from the NP group (*p* < 0.001). (b) MDA activity, ^∗∗∗^significant difference from the control group at *p* < 0.001, ^++^significant difference from the NP group (*p* < 0.001), and ^+++^significant difference from the NP group (*p* < 0.0001). (c) Total antioxidant capacity (TAC) activity, ^∗∗^significant difference vs. the control group at *p* < 0.001, ^+^significant difference from the NP group (*p* < 0.05), and ^++^significant difference from the NP group (*p* < 0.001). (d) SOD activity, ^∗∗^significant difference vs. the control group at *p* < 0.001, ^+^significant difference from the NP group (*p* < 0.05), ^++^significant difference from the NP group (*p* < 0.001). Bars represent mean ± SD (*n* = 4). NP: nonylphenol; MLT: melatonin.

**Figure 3:** Melatonin and nonylphenol did not change testosterone concentration. Comparison the level of testosterone in all experimental groups. Bars represent mean ± SD (*n* = 4).

**Figure 4:** Calibration chart. The ratio of the area under the curve to the concentration of NP *R*^2^ = 0/9957.

**Figure 5:** Nonylphenol HPLC spectrum. (a) Standard sample of NP (20 *μ*g/ml) and a sample of NP in the testicular tissue (200 mg) of the NP25 group. (b) The sample of NP in the testicular tissue (200 mg) of the NP25 group. (c) The sample of NP in serum of the NP+MLT20 group. (d) The sample of NP in serum of the NP+MLT10 group (*n* = 4). NP: nonylphenol; MLT: melatonin.

**Figure 6:** MLT improved histopathological changes induced by NP in the adult testis. Representative photomicrographs of the testis of first-generation adult male rats (H&E stain, ×40) (*n* = 4). Control group (a), MLT20 group (b), NP25 group (c), NP+MLT10 group (d), and NP+MLT20 group (e). (a) Shows normal tissue conditions in the control group; (b) normal tissue conditions and increased spermatozoa population in the MLT20 group; (c) hyperemia (right arrow), edema (down arrow), and vacuolar degeneration (arrow left) in the NP25 group; (d) hyperemia (arrow to the right) and vacuole degeneration (arrow to the left) in the NP+MLT10 group; and (e) normal tissue conditions in the NP+MLT20 group. NP: nonylphenol; MLT: melatonin.

**Table 1:** Mean (±SD) of nonylphenol concentration in groups (*n* = 4).

Groups	Concentration in tissues (ng/mg)	Concentration in serum (*μ*g/ml)
NP25	17/2 ± 3	N.D
NP+MLT10	14/1 ± 2	N.D
NP+MLT20	2/8 ± 0/21	N.D
MLT20	N.D	N.D

N.D: not detected; NP: nonylphenol; MLT: melatonin.

**Table 2:** Mean (±SD) of the diameter of seminiferous tubules, the thickness of the epithelium, the cross-sectional area of seminiferous tubules, the cross-sectional area of the epithelium of seminiferous tubules, number of seminiferous tubules, and count of spermatocytes and spermatogonia between groups (*n* = 4).

Groups	Cross-sectional area of seminiferous tubules (*μ*m^2^)	Cross-sectional area of seminiferous tubule epithelium (*μ*m^2^)	Thickness of epithelium (*μ*m)	Diameter of seminiferous tubules (*μ*m)	Number of spermatocytes	Number of spermatogonia	Number of seminiferous tubules
Control	42221.03 ± 2128.91^a^	29835.27 ± 1385.80^a^	93.23 ± 3.56^a^	258.20 ± 9.51^b^	80.00 ± 4.04^a^	80.24 ± 3.96^a^	11.14 ± 0.34^a^
NP	34283.80 ± 1612.15^b^	20507.37 ± 1093.34^b^	83.70 ± 2.56^b^	236.33 ± 6.84^b^	21.88 ± 0.99^b^	22.87 ± 1.25^b^	7.58 ± 0.25^b^
NP+MLT10	40149.90 ± 1796.04^a^	22835.60 ± 1076.96^b^	88.93 ± 1.813^a,b^	245.90 ± 5.21^b^	34.13 ± 2.81^a^	31.26 ± 2.56^b^	9.17 ± 0.24^a^
NP+ LT20	41218.63 ± 2453.05^a^	23790.10 ± 1102.77^b^	91.60 ± 3.94^a,b^	255.00 ± 7.61^b^	43.08 ± 4.34^a^	47.56 ± 4.51^a^	10.02 ± 0.35^a^
MLT20	42671.63 ± 1435.06^a^	31140.83 ± 1853.71^a^	92.90 ± 2.47^a^	251.87 ± 9.15^b^	84.89 ± 5.16^a^	78.76 ± 5.79^a^	10.79 ± 0.37^a^

Significant difference between the groups shown with different letters (a and b) (*p* < 0.05; one-way ANOVA followed by Duncan's test).

**Table 3:** Histopathological examination of the testicular tissue.

Groups	Edema	Hyperemia	Decrease spermatozoa	Vacuole degeneration
Control	—	—	—	—
NP	+	++	+	++
NP+MLT10	—	+	—	+
NP+MLT20	—	—	—	—
MLT20	—	—	—	—

## Data Availability

Upon request, data supporting the conclusion of our study are accessible by the corresponding author.
